# Acupoint Massage plus Recombinant Bovine Basic Fibroblast Growth Factor Ophthalmic Gel and Limbal Stem Cell Transplantation on Visual Quality, Corneal Refraction, and Aesthetic Outcome in Patients with Pterygium

**DOI:** 10.1155/2022/7103496

**Published:** 2022-06-14

**Authors:** Xiaoqin Zhang, Yu Wu

**Affiliations:** Department of Ophthalmology, People's Hospital of Lujiang County, Hefei, Anhui, China

## Abstract

**Objective:**

To investigate the clinical study of acupoint massage combined with recombinant bovine basic fibroblast growth factor (rbFGF) ophthalmic gel combined with limbal stem cell transplantation on visual quality, corneal refraction, and aesthetic outcome in patients with pterygium.

**Methods:**

Sixty patients with pterygium treated in People's Hospital of Lujiang County from March 2018 to May 2021 were randomized into the control group and the research group by the random number table method, with 30 cases in each group. The control group received rbFGF plus limbal stem cell transplantation. The research group was treated with acupoint massage additionally.

**Results:**

The total clinical effective rate in the study group was higher than that in the control group (*P* < 0.05); after treatment, the modulation transfer function (MTF) cutoff and Strehl ratio (SR) levels in the study group were significantly higher than those in the control group, and the tear film-related objective scatter index (TF-OSI) was significantly lower than that in the control group (*P* < 0.05); corneal horizontal curvature and corneal vertical curvature in the study group after treatment were significantly higher than those in the control group, and corneal astigmatism degree (CAD) levels were significantly lower than those in the control group (*P* < 0.05); the levels of the break-up time (BUT) and Schirmer test (SIT) in the study group were significantly higher after treatment, compared with the control group (*P* < 0.05); and the incidence of adverse manifestations in the study group was significantly lower than that in the control group (*P* < 0.05).

**Conclusion:**

Acupoint massage combined with rbFGF ophthalmic gel combined with limbal stem cell transplantation is effective in clinical treatment of pterygium.

## 1. Introduction

Pterygium is a chronic inflammatory disease caused by external stimuli and is a common disease in ophthalmology [1]. Its occurrence and development are ascribed to external environmental stimuli or genetics [2]. Corneal invasion can result in changes in corneal morphology or refractive abnormalities [3]. If not treated in time, pterygium will gradually expand, which will have a significant impact on the patient's corneal astigmatism and eye movement and even reduce the patient's visual acuity [4, 5]. The final treatment of pterygium should achieve the purpose of restoring vision, improving cosmetic effects, and reducing adverse reactions and postoperative recurrence rates. Pterygium excision combined with limbal stem cell transplantation for the treatment of simple pterygium is widely recognized, which can effectively reduce the recurrence rate after simple excision, but some patients still experience recurrence [6]. rbFGF can promote the proliferation of wound corneal epithelial cells and tissue regeneration and repair after surgery, restore the corneal surface, effectively prevent the invasion of fibrous tissue and conjunctival epithelium into the cornea, and reduce the chance of wound infection [7]. rbFGF ophthalmic gel can relieve the symptoms of eye pain, dryness, and foreign body sensation to a certain extent [8]. Acupoint massage to our knowledge can relieve postoperative eye and head pain [9]. Corneal limbal stem cell transplantation can be performed with the assistance of the limbus. The regeneration ability of stem cells can repair and reconstruct the corneal limbal epithelial fine tissue, which can quickly restore the ocular surface function of patients and achieve the purpose of treatment [10]. This study intends to explore the clinical treatment of pterygium with acupoint massage plus rbFGF ophthalmic gel.

## 2. Materials and Methods

### 2.1. General Information

Totally 60 patients with pterygium were randomized into the control group and the research group by the random number table method, with 30 cases in each group. The patients in the control group included 12 males and 18 females, aged 45–83 years, mean age (63.13 ± 8.31) years, disease duration 6-7 years, and mean duration (6.47 ± 0.51) years. The patients in the research group included 16 males and 14 females, aged 49–78 years, mean age (62.90 ± 8.48) years, disease duration 6-7 years, and mean disease duration (6.57 ± 0.50) years. The baseline clinical data such as gender, course of disease, and age were similar in the two groups of patients. The studies involving human participants were reviewed and approved by People's Hospital of Lujiang County, no. LJH9979.

### 2.2. Inclusion and Exclusion Criteria

#### 2.2.1. Inclusion Criteria

Inclusion criteria were as follows: aged between 18 and 70; with corneal stem cell transplantation; complicated with pterygium after operation, the head of pterygium invades the cornea or the inner edge of the cornea; and all patients were informed and able to cooperate with the study for treatment and signed an informed consent.

#### 2.2.2. Exclusion Criteria

Exclusion criteria were as follows: patients with ocular surface infectious diseases and other ocular diseases such as fundus diseases; patients with severe systemic immune system diseases and patients with severe dry eye syndrome; patients with severe allergic constitution; with serious diseases of the whole-body functional organs such as the heart, liver, brain, and kidney; and with the history of other ophthalmic medication.

### 2.3. Treatment Methods

The control group received limbal stem cell transplantation plus rbFGF. The research group was treated with acupoint massage additionally. All patients in the group received treatment for 30 days.

#### 2.3.1. Limbal Stem Cell Transplantation

The pterygium excision and corneal limbal stem cell transplantation was conducted as follows. (1) The conjunctiva sac was routinely cleaned, the eyelid and adjacent skin were disinfected, and 2% lidocaine was injected into the neck and body of pterygium for anesthesia. The pterygium head was held with dentified forceps. The pterygium head was dissected at a shallow layer of about 0.5 mm, which was separated to the limbus of the cornea, and the conjunctiva on both sides of pterygium was cut open. (2) The bulbar conjunctiva of the body was separated and bluntly separated from the sclera; then, the head and neck of pterygium were cutoff. (3) A conjunctiva flap of corresponding size was made in the bulbar conjunctiva above the temporal. The conjunctiva graft was laid in the sclera exposed area, and the 10-0 nylon thread was intermittently sutured in the shallow sclera.

#### 2.3.2. rbFGF Ophthalmic Gel

rbFGF ophthalmic gel (manufactured by Zhuhai Essex Biopharmaceutical Co., Ltd., approved by the national medicine 05171204), was used 4 times/d, 1-2 drops/time, twice a day.

#### 2.3.3. Acupoint Massage after Operation

Acupoint massage was performed, and the thumb was pressed on Fengchi, Neiguan, and Zanzhu points with a depth of about 0.5 cm, and acupoints were pressed for about 5 minutes, so that the patient felt sore, numb, distended, and painful, once every 6 hours, for a total of 4 times.

### 2.4. Observation Indicators

1. The clinical efficacy of the two groups of patients was analyzed and recorded. Cured: the corneal wounds of the patients were well covered, and the conjunctiva was flat and no congestion. Effective: the symptoms of the patients were improved. Recurrence: the conjunctival hyperemia was obvious, and neovascularization grew with proliferation of conjunctival fibrous tissue and invaded the cornea.
2. The improvement of visual quality [11] in the two groups before and after treatment was compared, including whether SR, TF-OSI, and MTF cutoff indexes increased or decreased
3. The corneal refractive status of the two groups of patients before and after treatment, including changes in CAD, corneal horizontal curvature, and corneal vertical curvature level, were compared and analyzed
4. The changes of tear film function [12] in the two groups before and after treatment, including the changes of BUT and SIT levels, were observed and compared
5. The influence of the two groups of patients on the cosmetic effect after treatment and the incidence of adverse manifestations such as subvalvular effusion, opacity of the transplanted flap, and congestion in the transplanted area were compared

### 2.5. Statistical Methods

SPSS 25.0 was used for data analysis. Measurement data in this study were analyzed by the *t*-test, and count data were compared using the *χ*^2^ test.*P* < 0.05 was considered statistically significant differences.

## 3. Results

### 3.1. Clinical Efficacy

The total clinical effective rate of the study group was 93.33%, which was significantly higher than that of the control group (70.00%) (*P* < 0.05), as given in Table 1.

### 3.2. Improvement of Visual Quality Parameters

There was no significant difference in SR, TF-OSI, and MTF cutoff between the two groups before treatment (*P* > 0.05); the levels of MTF cutoff, SR, and TF-OSI in the two groups after treatment were significantly improved, with higher MTF cutoff and SR and lower TF-OSI results in the study group compared with the control group (*P* < 0.05), as given in Table 2.

### 3.3. Corneal Refractive Status

There was no significant difference in CAD, corneal horizontal curvature, and corneal vertical curvature between the two groups before treatment (*P* > 0.05). Corneal vertical curvature and CAD level were significantly improved, and the corneal horizontal curvature and corneal vertical curvature in the study group were significantly higher than those in the control group, and the CAD level was significantly lower than that in the control group (*P* < 0.05), as given in Table 3.

### 3.4. Changes of Tear Film Function

There was no significant difference in the levels of BUT and SIT between the two groups before treatment (*P* > 0.05). The levels of BUT and SIT increased in the two groups after treatment, with higher results in the study group (*P* < 0.05), as given in Table 4.

### 3.5. Cosmetic Outcomes

After treatment, the incidence of adverse reactions in the study group was significantly lower than that in the control group (13.33% vs. 50.00%) (*P* < 0.05), as given in Table 5.

## 4. Discussion

Though the etiology of pterygium remains unclear etiology, the contributors such as genetic and environmental factors and chronic long-term stimuli such as dust, smoke, and sunlight have been identified [13, 14]. External stimuli lead to increased vascular permeability in the corner of the eye, resulting in a decrease in the proliferation of stem cell transplantation, a decreased ability to regulate differentiation, abnormal proliferation of ocular fibroblasts, and the formation of new blood vessels [15]. There is mild discomfort in the early stage of the disease, and it can cause astigmatism or visual impairment and even restrict the patient's eye movement. As the disease progresses, pterygium may have irritation symptoms when it enlarges, substantially interfering with the appearance and vision [16]. Treating the recurrence of pterygium remains a pressing issue. In recent years, limbal stem cell transplantation has yielded remarkable results, but the operation is complicated and has limitations [17]. Therefore, nonsurgical methods are desired for its treatment as a supplement to surgery. We hypothesize that the use of acupoint massage combined with rbFGF ophthalmic gel combined with limbal stem cell transplantation would produce a good prognosis.

In line with our hypotheses, after treatment, the levels of MTF cutoff and SR in the two groups increased, while the level of TF-OSI decreased, with higher MTF cutoff and SR and lower TF-OSI in the study group suggesting that the visual quality of the patients was improved and the tear film function was effectively restored. Some studies have also confirmed that Pterygium can impair visual quality, and pterygium excision can significantly improve visual acuity 6 months after surgery [18]. Also, in keeping with our hypotheses, the corneal horizontal curvature and corneal vertical curvature of the two groups were increased, and the CAD level was decreased. This would suggest that after surgery, the removal of pterygium reduces the occlusion effect, pupil astigmatism, and impact on corneal diopter, effectively relieves the pressure of the lesions on corneal tissue, improves the ocular surface structure, and minimizes the damage to the eye. In support of our findings, a prior study argued that pterygium excision has a remarkable astigmatism effect on the posterior surface of cornea, and the effect of astigmatism increased with age and higher preoperative posterior astigmatism [19]. Pterygium not only causes corneal irregularities, conjunctival congestion, and tear film changes but also has a significant impact on the ocular surface by directly changing the morphology of the meibomian gland, causing visible symptoms and potential signs of dysfunction [20]. After treatment, BUT and SIT levels in the two groups increased, and the study group was significantly higher than the control group, suggesting that the treatment can effectively improve the symptoms of dry eye and improve the function of the lacrimal gland. Additionally, the study group experienced lower incidence of adverse reactions and had a higher total clinical response rate. All these suggested that the combination of the three has good efficacy and safety profiles.

## 5. Conclusion

Acupoint massage combined with rbFGF ophthalmic gel combined with limbal stem cell transplantation in the treatment of pterygium relieves the pain of patients, regulates the abnormal ocular surface function of patients, and improves the visual quality, corneal refraction, and ocular, with good aesthetic outcome. It merits clinical promotion.

## Figures and Tables

**Table 1:** Comparison of clinical efficacy (*n* (%)).

Groups	Cured	Effective	Recurrence	Total
Control group (*n* = 30)	8 (26.67)	13 (43.33)	9 (30.00)	21 (70.00)
Study group (*n* = 30)	20 (66.67)	8 (26.67)	2 (6.67)	28 (93.33)
*χ* ^2^				5.46
*P*				0.02

**Table 2:** Improvement of visual quality parameter ($\bar{x}$ ± *s*).

Groups	SR		TF-OSI		MTF cutoff	
	Before	After	Before	After	Before	After
Control group (*n* = 30)	0.07 ± 0.04	0.13 ± 0.06	1.53 ± 0.14	0.65 ± 0.28	9.31 ± 1.25	19.58 ± 1.28
Study group (*n* = 30)	0.08 ± 0.04	0.18 ± 0.04	1.52 ± 0.13	0.50 ± 0.23	9.30 ± 1.26	20.47 ± 1.68
*t*	0.97	3.79	0.29	0.26	0.30	2.31
*P*	0.33	<0.001	0.77	0.02	0.98	0.02

**Table 3:** Comparison of corneal refractive status ($\bar{x}$ ± *s*).

Groups	CAD		CHC		CVC	
	Before	After	Before	After	Before	After
Control group (*n* = 30)	1.61 ± 0.14	0.58 ± 0.18	39.01 ± 5.24	45.24 ± 5.25	40.20 ± 4.35	43.19 ± 4.19
Study group (*n* = 30)	1.60 ± 0.16	0.47 ± 0.13	40.02 ± 5.16	47.82 ± 4.10	40.17 ± 4.23	47.24 ± 4.30
*t*	0.26	2.71	0.75	2.12	0.02	3.69
*P*	0.79	<0.001	0.45	0.03	0.97	<0.001

CAD, corneal astigmatism degree; CHC, corneal horizontal curvature; CVC, corneal vertical curvature.

**Table 4:** Comparative analysis of changes in tear film function ($\bar{x}$ ± *s*).

Groups	BUT (s)		SIT (mm/5 min)	
	Before	After	Before	After
Control group (*n* = 30)	9.51 ± 0.24	12.15 ± 1.29	12.25 ± 0.24	13.12 ± 0.14
Study group (*n* = 30)	9.50 ± 0.22	13.93 ± 1.26	12.23 ± 0.30	13.95 ± 0.32
*t*	0.16	5.40	0.28	13.01
*P*	0.86	<0.001	0.77	0.01

**Table 5:** Analysis and comparison of cosmetic effects (*n* (%)).

Groups	Subvalvular effusion	Opaque graft flap	Congestion in the transplant area	Adverse manifestations rate
Control group (*n* = 30)	4 (13.34)	4 (13.34)	7 (23.32)	15 (50.00)
Study group (*n* = 30)	2 (6.67)	1 (3.33)	1 (3.33)	4 (13.33)
*χ* ^2^				9.32
*P*				<0.001

## Data Availability

No data were used to support this study.
